# Day Surgery Scheduling and Optimization in Large Public Hospitals in China: A Three-Station Job Shop Scheduling Problem

**DOI:** 10.1155/2022/1149657

**Published:** 2022-07-30

**Authors:** Xue Bai, Wei Zhang, Li Luo, Hongsheng Ma, Ting Zhu

**Affiliations:** ^1^Institute of Hospital Management, West China Hospital, Sichuan University, Chengdu 610041, China; ^2^Department of Industry Engineering, Business School, Sichuan University, Chengdu 610041, China; ^3^Day Surgery Center, West China Hospital, Sichuan University, Chengdu 610041, China

## Abstract

Day surgery scheduling allocates hospital resources to day surgical cases and decides on the time to perform the surgeries in the day surgery center (DSC). Based on the day surgery service process of large public hospitals in China, we found that the service efficiency of the process depends on the utilization of hospital resources efficiently and could be optimized through day surgery scheduling. We described it as a flexible flow shop owing to the three-station nature of surgery. Allocating all types of hospital resources to the three stations and determining the length of time for each stage during surgery are crucial to improving the efficiency of DSC. This paper integrates a three-station job shop scheduling problem (JSSP) into the day surgery scheduling and optimization problem. The JSSP was formulated as a mixed-integer linear programming model, and the elicitation of the model for scheduling surgeries with different priorities in the DSC is discussed. The model illustrated a case study of the DSC within West China Hospital (WCH). Numerical experiments based on the genetic algorithm design were conducted. Compared to the other optimization strategies, we proposed that the three-station job shop scheduling strategy (TSJS) could not only improve the efficiency and reduce the waiting time of the patients of the DSC in large public hospitals in China but also allow for timely scheduling adjustments during the advent of emergency surgeries.

## 1. Introduction

The proportion of day surgery is steadily growing globally [1, 2], which has had a substantial positive economic and social impact on the medical service system. In the United States and other developed countries, day surgery accounts for more than 60% of all surgeries, and the types of day surgery cover almost all surgical departments [3]. Compared to other countries, day surgeries in China have only just begun. In West China Hospital (WCH), the operating room represents a bottleneck with more than 3 months of waiting time for the patients; some patients even wait for the day surgeries for more than 1 year; operating rooms scheduling should obviously develop targets for waiting time, cost reduction, and resource use improvement. The day surgery features a shorter waiting time and length of stay, lower medical expenses, and a higher hospital bed utilization rate. All of these advantages have prompted more crowded, large public hospitals in China to adopt the day surgery model. Currently, the WCH, reporting the highest proportion of day surgeries nationally, stands at only 23% [4]. Instead of establishing independent day surgery centers (DSCs) as in other countries, the WCH establishes internal DSCs and shared operating rooms for elective and urgent surgeries (Figure 1). To reduce the medical safety risk, we established strict admission criteria for the day surgery, such as the patient's age, and clinical pathway. Compared to elective surgery with several days staying in the hospital, day surgery patients only need to stay for one night. Typically, day surgeries are shorter, less complex, and less variable than inpatient surgeries.

Note that DSS, because both the day surgeries and elective surgeries are planned in advance and urgent surgeries cannot be planned in advance and need to be scheduled as soon as possible for higher priority, the day surgery scheduling (DSS) in WCH must deal with different types of cases, having different priorities and predictability. To control the flow of patients, the DSS decides on the resource assignment and sequence of the cases in a short-term time horizon. Obviously, it is more difficult to optimize the DSS in this internal DSC of WCH for different priority surgeries shared with the resources.

Based on the day surgery service process of WCH, we found that the patient flow passes through three stations (Figure 2). The first station is preoperative anesthesia, which is performed in the anesthesia preparation room (APR). The anesthesia time is mainly related to the types of cases. The second station is the surgery, which is completed in the operating room (OR) and includes the setup (preincision), surgery (incision), and cleanup (postincision). Furthermore, the duration of this stage is the total time taken to perform the three parts. The phases occupy the same resources, including surgeons and ORs. The surgical case setup and cleanup time are relatively fixed and depend on the type of surgery. The surgery time is related not only to the type of surgery but also to the surgeon. The third station is the anesthesia preparation, which is performed in the anesthesia recovery room (ARR), and the anesthesia resuscitation time is mainly related to the types of cases. Allocating the different kinds of resources to the three stations and scheduling surgical cases on allocated resources are two questions that the DSS addresses. DSS must deal with different types of cases, having different priorities and predictability.

We depict the DSS problem as a three-station JSSP according to the day surgery process. It formulates the JSSP as a mixed-integer linear programming (MILP) model and discusses the use of the model for scheduling surgeries with different priorities. The model illustrates a detailed example of the DSC of WCH, which completed a total of 19,830 surgeries in 2019. The surgery type and the number of available ORs and surgeons are determined 24 hours in advance. Using preliminary computational experiments with MATLAB, we meticulously gathered the DSS policy and complete surgery information, including when surgery starts and finishes in every station, which resources are needed, and when the resource is occupied and released. It not only can shorten the span of the whole process but also can reduce the time wasted in the OR. The most important point is that optimal scheduling can timely adjust the scheduling result when a high-priority surgery comes in and needs to share the operating rooms.

The contributions made in this paper are summarized as follows. First, we integrate a three-station job shop scheduling problem into the day surgery scheduling according to the patient flow of DSC. Second, we constructed a mathematical model considering the different kinds of resource constraints in day surgery that not only can reduce the waste time of ORs but also can meet the resource constraint of personnel (anesthesiologists, surgeons, and anesthesia resuscitation doctors) and facilities (APRs, ORs, and ARRs). Third, we propose a new strategy, TSJS, to ensure that emergency surgeries are scheduled after the earliest completed elective surgeries when emergency surgery needs to be shared with the operating rooms.

## 2. Literature Review

May et al. [5] divided surgery planning and scheduling into six categories: very long term, long term, medium term, short term, very short term, and contemporaneous according to the time framework. They analyzed the future research orientation from the aspects of capacity planning, process reengineering/redesign, surgical service portfolio, procedure duration estimation, schedule construction, schedule execution, monitoring, and control. van Oostrum et al. [6] proposed cyclic operating room schedules, so-called master surgical schedules (MSSs), to maximize the operation room utilization and level the requirements for subsequent hospital beds, such as wards and intensive care units. Cardoen et al. [7] noted that the study of surgery scheduling in an uncertain environment and the collaborative optimization of multiple resources would be the two main directions of the development of surgery scheduling. Xiang and Li [8] proposed and defined a short-term surgery scheduling problem to optimize OR management and reduce operation costs based on a survey of the OR operation in a typical hospital in China. Luo et al. [9] proposed a rolling horizon mixed-integer programming model for scheduling. Considering the day-to-day demand for surgery, they developed a nonrolling scheduling model (NRSM) and a rolling horizon scheduling model (RSM) to balance the occupancy time among operating rooms. Gür and Eren [10] presented a detailed analysis of 170 studies by reviewing the literature on recent research on OR scheduling and planning from 2000 to the present day. They categorized the studies in the literature according to patient characteristics, performance measures, solution techniques used in the research, the uncertainty of the problem, applicability of the research, and the planning strategy to be dealt with within the solution. Ansarifar et al. [11] formulated operating rooms considering several constraints, such as decision-making styles, multiple stages for surgeries, time windows for resources, and specialty and complexity of the surgery. They proposed an integrated fuzzy possibilistic–stochastic mathematical programming approach, considering some sources of uncertainty simultaneously. Wu et al. [12] proposed the joint problem of planning and scheduling patients in operating rooms on an operational level (weekly basis) with two objectives: maximizing the overall patients' satisfaction and minimizing the cost of overtime in operating rooms as well as the daily cost of operating rooms and recovery beds. Nasiri et al. [13] developed a fuzzy robust stochastic optimization approach to tackle the multiobjective surgery scheduling model. Umali et al. [14] aimed to assess operating room efficiency for resident-performed elective phacoemulsification surgeries performed under local anesthesia by measuring different key performance indicators and comparing this with international benchmark data. Hsu et al. [15] proposed scheduling of surgical operations across multiple operating rooms subject to the limited availability of anesthetists; they abstracted the problem into a theoretical server scheduling problem and formulated an integer programming model to construct a feasible operations schedule that has the minimum makespan. Calegari et al. [16] proposed a heuristic to sequence surgeries that considers both upstream and downstream resources required to perform them, such as surgical kits, postanesthesia care unit (PACU) beds, and surgical teams (surgeons, nurses, and anesthetists). Lin and Chou [17] studied the operating room scheduling problem of assigning a set of surgeries to several multifunctional operating rooms and constructed a mathematical model to assign surgeries to operating rooms within one week. Zhang and Su [18] formulated a new stochastic programming formulation to solve the dynamic scheduling problem in a given set of elective surgeries on the day of operation and presented a mathematical model to improve resource utilization as measured by surgeon waiting time and operation room idle time.

Although the benefits of efficient scheduling systems are publicized in many industrial applications, such as job shop scheduling (JSS) theory, which has provided theoretical guidance for high-efficiency production in the manufacturing industry, surgery scheduling literature with industrial applications is relatively scarce. Hsu et al. [19] proposed ASC surgical case scheduling as a two-stage no-wait flow shop. The first stage was the OR with surgeons as its main resources, and the second stage was the PACU with nurses. They proposed a heuristic approach that solved two subproblems interactively to minimize the number of PACU nurses and the makespan. Guinet and Chaabane [20] also modeled inpatient scheduling as a two-stage no-wait flow shop, but no solution approach was attempted. Klinkert and Klinkert [21] proposed a new surgical case scheduling approach that uses a novel extension of the job shop scheduling problem called the multimode blocking job shop (MMBJS). They formulated a mixed-integer linear programming problem and discussed the use of the MMBJS model for scheduling elective and add-on cases. Agrawal et al. [22] addressed the problem of finding an assignment of *n* surgeries to be performed in one of *m* parallel identical operating rooms (ORs), given that each surgery had a stochastic duration with a known mean and standard deviation. The objective was to minimize the maximum of the makespan of any OR.

Surgical scheduling problems were proved to be NP-hard, and heuristics were developed in these problems. Hans et al. [23] proposed various constructive heuristics and local search methods that use statistical information on surgery durations to exploit the portfolio effect and thereby to minimize the required slack. Roland et al. [24] introduced a genetic algorithm (GA) approach to heuristically solve the operating theatre planning optimization problem, and this method had been widely used in the study of surgical scheduling problems. An exact method, simulated annealing (SA), GA, an ant colony optimization (ACO) algorithm, and some new soft computing strategies were proposed in [25–29] to solve scheduling problems.

Finally, we are not aware of any literature on DSS in Chinese hospitals. Many papers focus on the OR when discussing the SCS. However, efficiency gains might be achieved by considering not only the OR but also its adjoining units. Indeed, there are strong interactions between the OR and pre- and postoperative facilities, as shown in the day surgery process. Most studies consider the use of only one resource (ORs or nurses) during any operation and not the simultaneous use of multiple resources. Some research [21, 30] considers various practical constraints of the surgery scheduling problem: regular opening hours, maximum overtime hours allowed by the labor legislation, surgeons' availability and the type of equipment available in each operating room, and so on. In this article, we considered constraints of the undetermined resources, matched the day surgery with various resources in different procedures of the day surgery based on the previous studies, and presented the optimized scheduling results in the JSSP model.

## 3. Model Formulation and Discussion

### 3.1. A Mixed-Integer Linear Programming Model for DSS

Jain and Meeran proposed that most of the extensions of job shop scheduling address only one or two practical aspects not covered in the classical job shop problem, for example, job shop scheduling with multiprocessors and flexible processors [31]. Klinkert and Klinkert [21] proposed a novel extension to the JS called MMBJS. Each job consists of a sequence of operations. The execution of an operation requires a set of resources (a mode); resources are not always available all the time while depending on the mode. Based on the research of Pham and Klinkert, we use the available time of different kinds of resources to optimize the day surgery scheduling instead of the mode. Scheduling the jobs means assigning the resources and determining the starting and leaving time for the objective function is minimized.

According to the day surgery flow in WCH, a case typically comprises three steps, corresponding to the preoperative, perioperative, and postoperative stages. The duration of every step is the total setup time, processing time, and cleanup time. The resources needed for performing a day surgery comprise personnel (anesthetists, surgeons, and anesthesia resuscitation doctors) as well as facilities (anesthesia preparation room (APR), operating room (OR), and anesthesia recovery room (ARR)). There is no buffer between resources so that if a job has finished an operation and the job's next operation cannot be started, the resources of the finished operation remain blocked until the next operation is started. We assume that the duration of the setup time and cleanup of each operation is fixed and known before the surgeries, and the APR, OR, and ARR—as the three kinds of resources required in the three operations—have an equal opening time. The processing time of the three operations will be affected by surgery types and personnel resources. We provide the surgical case (job) set with different types of day surgeries and surgeons and select jobs according to the day surgery requirements 24 hours in advance. Scheduling the jobs means assigning the resources and determining the starting and leaving times for each operation. The aim of DSS is to determine a schedule for a given set of day surgical cases that minimizes some objective function. In line with high resource utilization, the objective considered here involves the makespan. A schedule defines the processing steps of each case of the chosen resource, as well as the starting times and the leaving times.

The model is characterized by the following notations in Table 1.

The objective function is as follows:

1. To minimize the makespan, given by *x*_*τ*_, the operations are forced to start as early as possible by minimizing, as a second term with a small weight *α*, the sum of all starting times.

(1) $$\begin{array}{c} \text{Min}x_{\tau }+\alpha \sum_{r=1}^{R}\sum_{i=1}^{I}x_{J_{i}}^{r}. \end{array}$$

Constraints of the model are as follows:

(2) If resource *r* is assigned to *J* before resource *u*, the leaving time of operation *j* on resource *r* plus the processing time of operation *i* on resource *u* should be earlier than the leaving time of operation *i* under resource *u*;
  (2) $$\begin{array}{c} L_{J_{i}}^{u}-t_{J_{i_{dp}}}^{u}+H\left(1-\theta_{J}^{ru}\right)\geq L_{J_{j}}^{r},J\in ℑ,r,u\in R,r\neq u,i\neq j. \end{array}$$
(3) If surgery *J* is scheduled before surgery *Q* on the shared resource *r*, then a doctor (anesthetists, surgeons, and anesthesia resuscitation doctors) can only be assigned to one surgery at the same time;
  (3) $$\begin{array}{c} x_{Q_{i_{dp}}}^{r}\geq \left(x_{J_{i_{dp}}}^{r}+t_{i_{dp}}^{r}\right)-H\left(1-y_{JQ}^{r}\right),J,Q\in ℑ. \end{array}$$
(4) Resource *r* can only be assigned to one job at the same time;
  (4) $$\begin{array}{c} x_{Q_{i_{dp}}}^{r}\geq \left(x_{Ji_{dp}}^{r}+t_{i_{dp}}^{r}+t_{i}^{c}\right)-H\left(3-y_{JQ}^{r}-z_{J_{i}}^{r}-z_{Q_{i}}^{r}\right),JQ\in ℑ. \end{array}$$
(5) The processing time of the operation *i* of the day surgery *J* under resource *r* is between the starting time and the leaving time;
  (5) $$\begin{array}{c} L_{J_{i}}^{r}-x_{J_{i}}^{r}-t_{i_{dp}}^{r}z_{J_{i}}^{r}\geq 0;i\in I,r\in R_{i}. \end{array}$$
(6) The leaving time minus the starting time of the operation *i* of the day surgery *J* under resource *r* is smaller than the processing time plus the maximum waiting time allowed for operation *i* before it is moved to the next stage;
  (6) $$\begin{array}{c} L_{J_{i}}^{r}-x_{J_{i}}^{r}-t_{i_{dp}}^{r}z_{J_{i}}^{r}\leq b_{i};i\in I,r\in R_{i}. \end{array}$$
(7) When using the same resource *r*, the starting time of the operation *i* of the day surgery *Q* minus the leaving time of the operation *i* of the day surgery *J*, which is scheduled before the job *Q*, should be bigger than the sum of the preparation time of the job *J* and the cleanup time of the job *Q*;
  (7) $$\begin{array}{c} x_{Q_{i}}^{r}-L_{J_{i}}^{r}+H\left(2-z_{J_{i}}^{r}-z_{Q_{i}}^{r}\right)+H\left(1-y_{JQ}^{r}\right)\geq t_{i}^{c}+t_{i}^{s};J,Q\in I,J\neq Q,J<Q,r\in R \end{array}$$
(8) The starting time of the dummy operation *τ* minus the leaving time of the operation  *i* of the day surgery *J* under resource *r* should be longer than its cleanup time.
  (8) $$\begin{array}{c} x_{\tau }-L_{J_{i}}^{r}\geq t_{i}^{c};i\in I,r\in R_{i}. \end{array}$$
(9) The starting and leaving time of the operation should be non-negativity.

(9) $$\begin{array}{c} x_{J_{i}}^{r},L_{J_{i}}^{r},x_{\tau }\geq 0;i\in I,r\in R_{i}. \end{array}$$

### 3.2. Considering the Emergency Surgeries for DSS

Large Chinese public hospitals usually establish internal DSCs or shared operating rooms between elective and urgent surgeries. Based on the JSSP model and considering the impact of emergency surgery on DSS strategies, emergency surgery will be given the highest priority, but the time of arrival is uncertain. Many scholars have used the simulation method to study the law of emergency cases. Krajewski and Bossmeyer [32] proposed that the emergency complies with the normal distribution through statistical analysis and conducted research. Based on this research, Sinreich and Marmor [33] further studied the model of emergency patient arrival and comprehensively considered the impact of the type of patient, type of hospital, and length of time, signifying a normal distribution.

In this paper, we collected the emergency case data of the three types of bile duct surgery in WCH as the sample for statistical analysis. The statistical analysis also found that the arrival time in the day was subject to a normal distribution, which was consistent with that of existing studies. Therefore, this research simulates the normal distribution of emergency surgeries in a WCH based on real data and uses the normal distribution generator of MATLAB to produce emergency case requirements according to the normal distribution. As the aim is to explore the impact of emergency surgeries on the scheduling strategy of day surgeries, the process of statistical analysis will not be described.

In this model, the emergency surgeries will be scheduled after the earliest day surgery is completed, and all the day surgeries will be rescheduled in accordance with the original optimization of the scheduling strategy. This is different from the scheduling and optimization of the OR in WCH, where the emergency surgeries are given the highest priority and the day surgeries will be postponed successively and not rescheduled. In our model, the emergency surgeries and unscheduled day surgeries will be rescheduled again.

The model is characterized by the following notations in Table 2.

The objective function is as follows:

(10) To ensure that emergency surgeries can be scheduled as soon as possible, *βx*_*J*_*i*_^*E* ^_^*r*^ is the emergency surgery priority.

(10) $$\begin{array}{c} \text{Min}x_{\tau }+\alpha \overset{R}{\underset{r=1}{\sum }}\overset{I}{\underset{i=1}{\sum }}x_{J_{i}}^{r}+\beta x_{J_{i}^{E}}^{r}. \end{array}$$

Constraints of the model are as follows:

(11) The starting time of the emergency surgery is later than its arrival time;
  (11) $$\begin{array}{c} x_{J_{i}}^{r}\geq t_{J_{i}},J_{i}\in J_{i}^{E}. \end{array}$$
(12) The starting time of the emergency surgery is earlier than its latest start time. Because emergency surgery can only be scheduled after the ongoing elective day surgery is completed, it may exceed its latest start time, which requires the surgeon to take some action to help the patient extend the waiting period;
  (12) $$\begin{array}{c} x_{J_{i}}^{r}\leq t_{J_{i}}^{du},J_{i}\in J_{i}^{E}. \end{array}$$
(13) The starting time of the emergency surgery should be later than the available starting time of resource *r* when the day surgeries must be rescheduled.

(13) $$\begin{array}{c} x_{J_{i}}^{r}\geq e^{Rr},J_{i}\in J_{i}^{Rs}. \end{array}$$

### 3.3. Discussion

#### 3.3.1. Duration of the Day Surgery

Because of the short length of stay, WCH has specified the age range of the day surgery patients and surgical types and conducted medical procedures following the clinical pathway regulation, ensuring quality and safety of care for patients. Compared to elective surgery, the durations of the day surgery encompass less variability, and the setup time and cleanup time are relatively fixed and depend on the type of surgery. We assume that the same type of surgery has the same setup time and cleanup time. However, the processing time relates not only to the type of surgery but also to the surgeon's experience and techniques. Based on the analysis of data from 2019 to 2021 on biliary tract surgery for WCH, we assumed that all surgical procedures are known in this model and used the average time as the parameter in our computational study. Of course, if the dynamic changes and randomness are taken into consideration, the study will be more realistic and more complex.

#### 3.3.2. Planning Horizon

Foreign day surgeries have a longer planning horizon and are scheduled a few months ahead, closely related to the perfect surgical appointment mechanism and the medical insurance system. Therefore, the requirements will be reported to the hospital very early, enabling the hospital to make an early schedule. However, owing to incomplete surgical appointment mechanisms operationalized in China and the difference in the medical insurance system from foreign counterparts, day surgery can be included in the medical insurance reimbursement plan only after the preoperative examination is conducted for 21 days. This short planning horizon brings some problems, such as difficulty in optimizing the surgery scheduling. Moreover, the appointment center's work will be piled in the previous day because of a lack of long-term planning. Nevertheless, the short planning horizon has some advantages, including the dynamic and real-time adjustment of the surgery. Taking the above factors into consideration and based on the practices of WCH, we still set a 1-day planning horizon.

## 4. Computational Study

### 4.1. Genetic Algorithm

According to the three-station characteristics of DSS, we proposed a two-layer three-stage gene coding method as follows:

1. The length of the chromosome *l*=3*∗n*; *n* is the number of surgeries to be performed; and each day surgery has 3 procedures.
2. The code of the first layer represents the three procedures of the day surgery, which consists of three identical and randomly generated surgical sequence groups.
3. The code of the second layer represents the three types of rooms, and each code corresponds to a random sequence of room numbers. The three procedures of the surgery are randomly assigned to three types of rooms.

The following is an example of the chromosome (Figure 3): if there are three day surgeries: 1, 2, 3; two anesthesia preparation rooms (APR): 1, 2; two operating rooms (OR): 3, 4; two anesthesia recovery rooms (ARR) 5, 6; we use the two-layer three-stage gene coding method, and the chromosome coding is as follows:

The population size of the genetic algorithm (GA) is 30; the maximum algebra is 400; the crossover probability is 0.8; and the mutation probability is 0.3. We adopted roulette in the GA.

### 4.2. An Example of WCH

Considering the volume of the day surgery cases in the WCH, we selected the biliary tract surgery of DSC in WCH as a numerical example and conducted the schedule of day ORs.

#### 4.2.1. Types of Day Surgery

There are many types of day surgery in WCH, but laparoscopic cholecystectomy, cholecystectomy, and common bile duct exploration T-tube drainage account for more than 80% of the department's day surgeries. Therefore, we take these three kinds of surgery as the scheduling surgical types. Each surgery included preoperative anesthesia, surgery, and anesthesia resuscitation. Meanwhile, each operation also includes the setup time, processing time, and cleanup time.

#### 4.2.2. Types of Personnel Resources

According to the process of the day surgery, the personnel type involved in surgery implementation concerning the three processes includes anesthesiologists, surgeons, and anesthesia resuscitation doctors. We consider the example of DSC in WCH with three anesthesiologists, six surgeons, and three anesthesia resuscitation doctors. The corresponding matrix relation between the personnel and the type of surgery is exhibited in Table 3.

#### 4.2.3. Types of Facility Resources

The surgery is divided into three categories based on different facility resources (rooms) required–APRs, ORs, and ARRs; the number for each type of room is set as 4. We assume that these four rooms are available for three types of surgeries.

#### 4.2.4. Time Parameter

The duration of every operation equals the sum of setup time, processing time, and cleanup time. We assume that the setup time and cleanup time for operations are 30 minutes and 20 minutes, respectively. Table 3 shows three types of day surgeries planned to be performed and the information on processing time with assigned personnel in the three operations.

The processing time of anesthesia (Operation 1) and anesthesia resuscitation (Operation 3) mainly depends on the type of surgery and the specific parameters based on the actual statistical results of biliary surgery in WCH. The processing time of the surgery (Operation 2) depends on both the surgical type and the surgeons. The value at the intersection of surgical type and the surgeons is the processing time of this surgeon when conducting this type of surgery. If there is no specific value, it means that the surgeon does not perform this kind of surgery. According to the surgery requirements of surgeons and the parameter settings in Table 3, we can obtain the processing times of the day surgical cases.

### 4.3. Surgical Cases

#### 4.3.1. Day Surgeries

Surgery scheduling in WCH is performed 24 hours in advance. Consequently, the surgeons must put forward their surgery requirements to the DSC one day before patient admission.  Table 4 shows the surgical cases planned to be performed the next day, with information on the surgical type and the assigned doctors. There are six anesthesiologists {*A*_1_, *A*_2_, *A*_3_, *A*_4_, *A*_5_, *A*_6_}, three surgeons {*S*_1,_*S*_2,_*S*_3,_}, and three anesthesia resuscitation doctors {*D*_1,_*D*_2,_*D*_3,_} to schedule the three kinds of surgery. Each kind of day surgery (*d*) is performed by one anesthesiologist, one surgeon, and one anesthesia resuscitation doctor.

The actual data of the surgical requirements in the table are converted to the parameter table used for the scheduling model, as shown in Table 5.

#### 4.3.2. Emergency Surgeries

Based on the statistical analysis of the arrival times of emergency hepatobiliary surgery in the WCH, it is found that the arrival times follow the normal distribution: *N*(*μ*, *σ*^2^)(*μ*=1002.62, *σ*^2^=295.23). We use the MATLAB normal distribution generator to produce two emergency surgeries. The arrival times are 184 minutes and 250 minutes (calculated from 8:00 am).  Table 6 shows the information on the two arriving emergency surgeries to be performed.

The information of the simulated emergency surgeries was converted into the parameter table for the scheduling model, as shown in Table 7.

### 4.4. Calculation Results

#### 4.4.1. Scheduling Strategy of Day Surgery

Based on previous studies, we proposed the GA running the JSSP model on MATLAB and conducted the results denoting the best convergence effect at 30 seconds. The surgery sequencing strategy of each room is as shown in Table 8.

We can calculate the starting time of each process of the operations (set initial time as 0; Table 9).  Figure 4 shows the corresponding Gantt chart.

The calculation target value is 790.0149 minutes, and the population evolution figure is shown in Figure 5.

We can see from the above figure that the optimal individual appears at generation 120, and this individual remains optimal until generation 250. Therefore, generation 120 is the result we are seeking.

Monte Carlo simulation was carried out 300 times in our study. The distribution fitter toolbox of MATLAB was used to fit and observe the obtained data. We found that the results follow a normal distribution. According to the probability density and cumulative probability graph, the fitting effect was very good (Figure 6). The 95% confidence interval fitting results are as follows: the mean is 853.8198; the standard deviation is 31.0198; the confidence interval is [850.2954, 857.3442]; and the standard deviation of the confidence interval is [28.7203, 33.7226].

#### 4.4.2. Surgery Scheduling Strategy considering Emergency Surgeries

We proposed the genetic algorithm run the JSSP model on MATLAB and conducted the results denoting the best convergence effect at 30 seconds. The surgery sequencing strategy of each room is shown in Table 10.

We can calculate the starting time of each process of the operations (set initial time as 0; Table 11).  Figure 7 shows the corresponding Gantt chart.

The target value of the calculation is 2,480 minutes, and the population of the evolution figure is shown in Figure 8.

We can see from Figure 8 that the optimal individual appears at generation 60, and this individual remains optimal until generation 200.  Table 12 shows the emergency cases.

The emergency surgery 16 and 17 arrival times are 184 minutes and 250 minutes, respectively. According to the scheduling results of the JSSP model considering the emergency surgeries, both surgery 16 and surgery 17 are scheduled after the earliest completed elective surgeries with more than 60 min waiting time, so the surgeon should take protective measures during this period to increase the patients' waiting time. The scheduling of day surgeries will remain unchanged until the arrival of emergency surgeries; otherwise, rescheduling will be conducted together with the remaining day surgeries.

When one emergency surgery arrives, we obtain the optimal elective surgeries scheduling result. Considering the second emergency surgery arriving at 250 minutes, we rearranged the remaining surgeries dynamically. Monte Carlo simulation was carried out 300 times, and the fitting effect was also very good (Figure 9). The 95% confidence interval fitting results are as follows: the mean is 2337.53, the standard deviation is 251.2624, the confidence interval is [2311.982, 2363.078], and the standard deviation of the confidence interval is [234.4535, 270.6876].

### 4.5. Comparison of Optimization Strategies

#### 4.5.1. Comparison of Four Optimization Strategies

According to the three-station surgery flow in the DSC of WCH, we proposed the three-station job shop scheduling strategy (TSJS) for the day surgery scheduling and optimization problem. The following are the two components of the TSJS:

- The first component is emergency surgery, which has the highest priority, and needs to be scheduled after the earliest day surgery is completed
- The second component is dynamic ranking that is conducted with the goal of minimizing the total operating time of the remaining elective day surgeries.

If we do not consider emergency surgeries, we only need to use the second component of the TSJS. There are three scheduling strategies in the DSC of WCH: the first strategy is scheduling the surgeries according to the arrival time of the patients, we call it the first come first service (FCFS); the second strategy is to consider the surgeon's preference, some surgeons prefer to finish the long time surgeries before the short time surgeries, we call it longest processing time first (LPT); and the third strategy is to arrange the short time surgeries before the long time surgeries, we call it shortest processing time first (SPT). In order to compare the TSJS with the other scheduling strategies, we adopt random coding of the surgical procedures of the first layer based on the FCFS, LPT, and SPT, and the coding method of the second layer remains unchanged. Monte Carlo simulation was carried out 300 times in every strategy. By plotting the boxplot (Figure 10), it can be found that the proposed TSJS has the shortest average time and the smallest discrete degree.

#### 4.5.2. Comparison of Three Optimization Strategies considering Emergency Surgeries

If we consider emergency surgeries, we need to use the two components of the TSJS. There are two scheduling strategies based on the first component of the TSJS: the first strategy is scheduling the emergency surgeries first in the available rooms, the rooms were randomly assigned to the emergency surgeries, the left surgeries in the rooms occupied by emergency surgeries were postponed, and the order of the remaining surgeries and rooms remained unchanged; we call it randomly assigned operating rooms (ROR). The second strategy is scheduling the emergency surgeries first in the available rooms. Rooms are allocated according to the available time of the room closest to the emergency surgery. The remaining surgeries in the rooms occupied by emergency surgeries were postponed, and the order of the remaining surgeries and rooms remained unchanged, which we call assigned operating rooms (AOR). Monte Carlo simulation was carried out 300 times in every strategy. By plotting the boxplot (Figure 11), it can be found that the proposed TSJS has the shortest average time and the smallest discrete degree.

According to the results of the four strategies comparison, we found that the ROR takes the longest time after the arrival of emergency surgeries, leading to the cost of the DSC increasing. The AOR is better than the ROR, and the TSJS can ensure the shortest total makespan time, which proves that the TSJS is effective.

#### 4.5.3. Impact of Patient Waiting Time

Based on the comparative analysis of the previous strategies, we found that whether emergency surgeries were considered, the first component makes a key contribution to the TSJS. To determine the influence of the different strategies on patients' waiting time, we calculated the patients' waiting time under the different strategies and adopted the Monte Carlo simulation 300 times. Through plotting the boxplot (Figures 12 and 13), it can be found that patients' waiting time was significantly reduced by the TSJS.

#### 4.5.4. Impact of Operating Room Occupancy Time Equilibrium Index

In addition to the waiting time of patients, we also need to know the impact of different strategies on the balance of room utilization. Unbalanced operating room utilization will lead to an increase in DSC management costs. We define the operating room occupancy time equilibrium index as follows: utilization rate of each operating room = operating room usage time/operating room opening time. The equilibrium index is the variance of the utilization rate of all operating rooms. We adopted the Monte Carlo simulation 300 times and plotted the boxplot (Figures 14 and 15). It can be found that the equilibrium index of the room occupancy time was significantly reduced by the TSJS.

## 5. Conclusion

This paper identifies and analyzes the DSS problem in large public hospitals in China. We describe the day surgery process as a three-station JSSP, including scheduling day surgeries and emergency surgeries. Comparing the TSJS with the other scheduling strategies of the WCH, the JSSP model not only can reduce the makespan of the service time of ORs but also can meet the resource constraints of personnel (anesthesiologists, surgeons, and anesthesia resuscitation doctors) and facilities (APRs, ORs, and ARRs). Urgent surgeries are also taken into consideration. DSS should take a holistic view of all activities and resource constraints in the OR suite instead of focusing on only an individual stage, which is used in the DSC management in the WCH.

The paper points out the importance of connecting day surgical stages in scheduling and coordinating multiple resources during any surgical step in the hospital. By further refining the day surgery procedure, the JSSP model dispatches the resources involved in the various processes of the surgery. The switching time is reduced owing to the subdivision of the surgery process, resulting in an increase in OR utilization. This can also benefit the management of anesthesiologists, surgeons, anesthesia resuscitation doctors, and other hospital resources. Surgeons can go to the corresponding location to perform the surgery after finishing the preparation, without waiting for the switching of the surgery, which not only catalyzes the efficiency of the operation room management but also promotes the standardization of the surgery process. The results of this study show that the JSSP model is more suitable for the efficient management of DSCs in large public hospitals [34].

Although this study considered a variety of resource constraints based on the day surgery service process implemented in China, there are still some shortcomings, which need further research:

1. The three-stage JSSP model for DSS and optimization is a deterministic model, which means that the duration of a certain surgery conducted by the surgeon is already determined. However, in practice, the time of surgery is often uncertain. Therefore, considering the uncertainty of operation time is necessary for the model (including emergency surgery) to ensure that the DSS optimization strategy is more realistic.
2. Multidimensional uncertainty is a special property in the DSS and optimization problem, meaning that many more factors must be considered in the surgery scheduling process. Although this research has taken into account anesthesiologists, surgeons, anesthesia resuscitation doctors, APR, OR, and ARR, factors such as bed, ICU, and medical technical inspections, which have a significant impact on OR scheduling, have not yet been considered. Therefore, further investigation of factors that influence DSS and optimization will inevitably make the research problem more complex but more valuable as well.
3. The complexity, frequency, and large solution size of DSS and optimization make it difficult to rely on manual input. We must develop an interoperable hospital OR scheduling management system that provides the needed parameters from the operating system and conducts automatic calculations necessary for achieving an efficient and accurate plan. It is important to study how to install the results of this research into the management system of the hospital ORs, forming a practical management tool.

## Figures and Tables

**Figure 1:** The day surgery service process of West China hospital.

**Figure 2:** Three stations of the day surgery center of WCH.

**Figure 3:** An example of the chromosome.

**Figure 4:** Example Gantt chart.

**Figure 5:** Population evolution of the scheduling strategy of day surgery.

**Figure 6:** Normal distribution fitting diagram.

**Figure 7:** Example Gantt chart considering emergency surgeries.

**Figure 8:** Population evolution considering emergency surgeries.

**Figure 9:** Normal distribution fitting diagram considering emergency surgeries.

**Figure 10:** Boxplot of the four strategies.

**Figure 11:** Boxplot of the three strategies considering emergency surgeries.

**Figure 12:** Comparison of patients' total waiting time under the four strategies.

**Figure 13:** Comparison of patients' total waiting time under the three strategies considering Emergency Surgeries.

**Figure 14:** Operating rooms occupancy time equilibrium index.

**Figure 15:** Operating rooms occupancy time equilibrium index considering emergency surgeries.

**Table 1:** Parameters and descriptions.

Parameter	Description
*R*	Set of facility resources
*I*	Set of operations
*P*	Set of personnel resources
*D*	Set of day surgery types
*ℑ*	Set of jobs
*R*_*i*_	Set of facility resources used by the operation *i*, *i* ∈ *I*
*t*_*i*_*dp*__^*r*^	The processing time of the operation *i* under resource *R*_*i*_^*r*^
*t*_*i*_^*s*^	The setup time of operation *i* ∈ *I*
*t*_*i*_^*c*^	The cleanup time of operation *i* ∈ *I*
*b*_*i*_	The maximum waiting time allowed for operation *i* ∈ *I* before it is moved to the next stage
*e* ^*r*^	The available starting time of the resource *r* ∈ *R*_*i*_
*f* ^*r*^	The available ending time of the resource *r* ∈ *R*_*i*_
*H*	Huge number
*α*	Very small weight factor
*τ*	Dummy operation of zero duration, *τ* is after all operations
*J*_*i*_	Job to which operation *i* ∈ *I* belongs to
*i*_*dp*_	Operation *i* processed by surgeon *p*, belonging to type *d* of surgery *d* ∈ *D*, *p* ∈ *P*

Decision variables	

$z_{J_{i}}^{r}=\left\{\begin{array}{cc} 1, & \text{if resource }r\text{ is assigned to operation }i\text{ of the day surgery }J\\ \text{0,} & \text{otherwise} \end{array}\right.,\;i\in I,r\in R_{i}$	
$\theta_{J}^{ru}=\left\{\begin{array}{cc} 1, & \text{ if resource r is assigned to day surgery }J\text{ before the resource }u\\ 0, & \text{otherwise} \end{array}\right.,\;r,u\in R_{i},r<u,J\in ℑ$	
$y_{JQ}^{r}=\left\{\begin{array}{cc} 1, & \text{if surgery }J\text{ is scheduled before surgery }Q\text{ on the shared resource }r\\ 0, & \text{otherwise} \end{array}\right.,\;J,Q\in ℑ,J<Q,r\in R$	
*x*_*J*_*i*__^*r*^	Starting time of operation *i* of the day surgery *J* under resource *r*
*L*_*J*_*i*__^*r*^	Leaving time of operation *i* of the day surgery *J* under resource *r*
*x*_*τ*_	Starting time of dummy operation *τ*

**Table 2:** Parameters and descriptions used in the DSS model considering the emergency surgeries.

Parameter	Description
*J*_*i*_^*S*^	Day surgeries that have been scheduled before the arrival of emergency surgeries
*J*_*i*_^*E*^	Set of emergency surgeries
*J*_*i*_^*RS*^	Day surgeries that must be rescheduled after the arrival of emergency surgeries
*t*_*J*_*i*__	Arrival time of emergency surgery *J*_*i*_ ∈ *J*_*i*_^*E*^
*t*_*J*_*i*__^*du*^	The latest start time of emergency surgery
*e* ^*Rr*^	The available starting time of resource *r* when the day surgeries must be rescheduled
*β*	Priority parameter of emergency surgery

Decision variables	
*x*_*J*_*i*__^*r*^	Starting time of operation *i* of the emergency surgery *J* on resource *r*, *J*_*i*_ ∈ *J*_*i*_^*E*^
*L*_*J*_*i*__^*r*^	Leaving time of operation *i* of the emergency surgery *J* on resource *r*, *J*_*i*_ ∈ *J*_*i*_^*E*^

**Table 3:** The processing times of the three surgery operations (min).

Surgery type (*d*)	Personnel (*p*)												
	Operation 1 (anesthesiologists)			Operation 2 (surgeons)						Operation 3 (anesthesia resuscitation doctors)			
	1	2	3	1	2	3	4	5	6		1	2	3
1	30	40	35	80	80	70	90	—	60		40	40	40
2	60	80	70	—	140	130	110	150	—		50	50	50
3	75	70	65	210	190	160	150	190	—		60	60	60

**Table 4:** Information table of surgical cases.

Types of day surgery (*i*_*dp*_)	Anesthesiologists (*A*_*i*_)	Surgeons (*S*_*i*_)	Anesthesia resuscitation doctors (*D*_*i*_)
Laparoscopic cholecystectomy	6	1	1
Laparoscopic cholecystectomy	6	2	2
Laparoscopic cholecystectomy	2	3	3
Common bile duct exploration T-tube drainage	2	3	3
Common bile duct exploration T-tube drainage	2	2	2
Common bile duct exploration T-tube drainage	5	1	1
Cholecystectomy	5	2	2
Cholecystectomy	4	3	3
Laparoscopic cholecystectomy	1	3	3
Laparoscopic cholecystectomy	1	1	1
Cholecystectomy	4	1	1
Cholecystectomy	4	2	2
Common bile duct exploration T-tube drainage	1	3	3
Laparoscopic cholecystectomy	3	2	2
Common bile duct exploration T-tube drainage	3	2	2

**Table 5:** Surgical cases by type and the parameter table.

Job number (surgery number)	Surgery type number (*d*)	Processing time (min)		
		Operation 1 (anesthesia)	Operation 2 (surgery)	Operation 3 (anesthesia recovery)
1	1	30	60	40
2	1	40	60	40
3	1	35	80	40
4	3	65	190	60
5	3	70	190	60
6	3	75	190	60
7	2	80	150	50
8	2	70	110	50
9	1	35	80	40
10	1	30	80	40
11	2	60	110	50
12	2	80	110	50
13	3	65	210	60
14	1	40	70	40
15	3	70	160	60

**Table 6:** Emergency surgeries information table.

Types of emergency surgery	Anesthesiologists	Surgeons	Anesthesia resuscitation doctors
Laparoscopic cholecystectomy	1	6	2
Common bile duct exploration T-tube drainage	2	2	3

**Table 7:** Emergency surgeries parameter table.

Job number (surgery number)	Surgery type number (*d*)	Processing time (min)		
		Operation 1 (anesthesia)	Operation 2 (surgery)	Operation 3 (anesthesia recovery)
16	1	30	60	40
17	3	70	190	60

**Table 8:** Strategy table of the day surgery sequencing.

Room number	Day surgery number and sequence					
1	11	5	2	9	0	0
2	1	15	13	4	0	0
3	10	3	8	12	0	0
4	14	7	6	0	0	0
5	14	7	8	12	0	0
6	1	15	13	9	0	0
7	11	5	4	0	0	0
8	10	3	2	6	0	0
9	10	11	5	6	0	0
10	3	7	2	12	0	0
11	14	8	13	9	0	0
12	1	15	4	0	0	0

**Table 9:** Starting timetable of each process of the three operations.

Surgery number	Anesthesia (min)	Surgery (min)	Anesthesia recovery (min)
1	30	60	120
2	350	400	460
3	145	190	270
4	460	525	715
5	200	280	470
6	425	510	700
7	120	210	360
8	330	410	520
9	625	670	750
10	30	60	140
11	50	120	230
12	480	570	680
13	335	410	620
14	30	70	140
15	110	180	340

**Table 10:** Surgery scheduling strategy table considering emergency surgeries.

Room number	Day surgery number and sequence
1	11 5 **17** 12 9 0 0
2	1 15 13 6 0 0 0
3	10 3 **16** 8 4 0 0
4	14 7 2 0 0 0 0
5	14 7 13 4 0 0 0
6	1 15 **17** 12 0 0 0
7	11 5 8 9 0 0 0
8	10 3 **16** 2 6 0 0
9	10 11 5 **17** 9 0 0
10	3 7 13 12 0 0 0
11	14 **16** 0 0 0 0 0
12	1 15 2 8 6 4 0

The significance of bold values given in Table 10 are the emergency surgeries and the sequence.

**Table 11:** Starting timetable considering emergency surgeries.

Surgery number	Anesthesia (min)	Surgery (min)	Anesthesia recovery (min)
1	30	60	120
2	380	430	490
3	145	190	270
4	595	670	860
5	200	280	470
6	460	540	30
7	120	210	360
8	440	520	630
9	760	795	875
10	30	60	140
11	50	120	230
12	620	710	820
13	335	410	620
14	30	70	140
15	110	180	340
**16** (Emergency surgery)	280	320	380
**17** (emergency surgery)	390	470	660

The significance of bold values given in table 11 are the emergency surgeries and the starting time of each process.

**Table 12:** Emergency surgery timetable.

Emergency surgery number	Arrival time (min)	Starting time of anesthesia (min)	Waiting time (min)
16	184	250	66
17	250	360	110

## Data Availability

The data used to support the findings of this article are restricted by West China Hospital to protect patient privacy and avoid legal and ethical risks. Data are available from West China Hospital for researchers who meet the criteria for accessing confidential data.
